The article "Analysis of Maternal and Neonatal Outcome of Patients with Preterm Prelabor Rupture of Membranes" was published in 2022. Journal: J Healthc Eng.

# Analysis of Maternal and Neonatal Outcome of Patients with Preterm Prelabor Rupture of Membranes

**DOI:** 10.1155/2022/8705005

**Published:** 2022-03-14

**Authors:** Chunmei Yan, Xiaohui Deng, Fanzhen Hong

**Affiliations:** ^1^Center for Reproductive Medicine, Department of Obstetrics and Gynecology, Qilu Hospital, Cheeloo College of Medicine, Shandong University, Jinan, Shandong 250012, China; ^2^Department of Obstetrics, The Second Hospital of Shandong University, Jinan, Shandong, 250033, China

## Abstract

**Background:**

Preterm prelabor rupture of membranes (PPROM) increases risk of maternal and neonatal diseases. Expectant treatment is one major treatment for PPROM patients, but it raises concerns on infection. Currently, the optimal delivery time for PPROM patients is still unclear, and there are various outcomes for the patients with PPROM. Previous studies conducted to analyze the pregnancy outcome showed inconsistent results. The purpose of this study is to retrospectively analyze the maternal and neonatal outcomes for comparison among different latency periods of patients with PPROM at a university hospital in China.

**Method:**

This was a retrospective study. We divided all patients with PPROM into four groups according to gestational weeks, namely, group A (GA 24–27^+6^), group B (GA 28–31^+6^), group C (GA 32–33^+6^), and group *D* (GA34-36^+6^). The maternal and neonatal outcomes of each group were observed, respectively. Groups B and C were separately divided into two subgroups according to the median latency period of each group, namely, B1, B2, C1, and C2. Then, the differences of pregnancy outcomes between B1 and B2, C1 and C2, were compared, respectively. A *p* value < 0.05 was considered statistically significant.

**Result:**

Group A: the common maternal and neonatal complications were the increased infection index before labour, neonatal hyperbilirubinemia and neonatal respiratory distress syndrome. Groups B, C, and D: the common maternal and neonatal complications were the increased infection index before labour, fetal distress, neonatal pneumonia, neonatal hyperbilirubinemia, and patent foramen ovale. Comparison of pregnancy outcome between group B1 and group B2 showed higher incidence rate of increased infection index before labour, lower incidence rate of respiratory distress syndrome, electrolyte disturbance, and premature brain in group B2 than those in group B1. Comparison of pregnancy outcome between group C1 and group C2 showed the higher incidence of increased infection index before labour, bigger birth weight, and shorter hospital stay in group C2 than those in group C1.

**Conclusion:**

Increased infection index before labour was common maternal complication in four groups. Neonatal hyperbilirubinemia and neonatal pneumonia were top neonatal complications in four groups. The prolongation of latency period was beneficial to newborns of patients with gestational week at 28–31^+6^ weeks, while it did not benefit those with gestational week beyond 32 weeks.

## 1. Introduction

Preterm prelabor rupture of membranes (PPROM) is defined as the membrane rupture before the onset of labor that occurs before 37 weeks of gestation [1]. PPROM accompanies in approximately 3% of pregnancies and increases the risk of maternal and neonatal diseases [2–5].

Various epidemiological and clinical factors are considered to be related to PPROM, such as maternal reproductive tract infection, obstetric complications, behavioral factors, environmental changes, and fetal endocrine signals [6–8]. The main cause of perinatal and neonatal mortality is preterm birth, of which 40% is caused by PPROM [9]. Consequently, expectant treatment is an important treatment for patients with PPROM. However, prolonged latency period increases the risk of ascending reproductive tract infection, which might lead to intrauterine infection [10]. Obstetrical strategies to treat patients with PPROM remain controversial, and the optimal delivery time is unclear [1], which depends on an evaluation of the risks and benefits of attempted pregnancy prolongation compared with expeditious delivery [11]. Due to the different variety of expectant treatment and different quality of medical care, the pregnancy outcomes of patients with PPROM are different [12–15]. In previous studies, there is a lack of comprehensive observations on maternal and neonatal complications as well as the consideration of grouping patients. This study aimed to retrospectively analyze the pregnancy outcome of patients with PPROM at a university hospital located in northern China. Patients with PPROM in this study were grouped based on the gestational age, and their all maternal and neonatal complications were observed, screened, and analysed.

## 2. Methods

### 2.1. Study Design

Permission by the Ethics Committee of the Second Hospital of Shandong University was obtained.

This was a retrospective study. We divided all patients with PPROM into four groups based on gestational weeks, namely, group A (GA 24–27^+6^), group B (GA 28–31^+6^), group C (GA 32–33^+6^), and group *D* (GA34-36^+6^). The maternal and neonatal outcomes of each group were observed, respectively. The median latency period of group B was 4 days. Based on the median latency period, group B was divided into two groups B1 (latency period ≤4 days) and B2 (latency period >4 days). Similarly, group C was also divided into two groups according to its median latency period C1 (latency period ≤3 days) and C2 (latency period >3 days). Then, the difference of pregnancy outcome between B1 and B2, C1 and C2, was compared, respectively. Maternal outcome indicators included cesarean section rate, increased infection index before labour, uterine atony, and postpartum hemorrhage. Neonatal outcome indicators included birth weight, neonatal asphyxia, and admission to neonatal care unit (NICU).

Inclusion criteria: all patients with prelabor rupture of membranes between 24 and 36^+6^ gestational weeks were included who were admitted to the obstetrical department in the Second Hospital of Shandong University, between January 1, 2016, and December 31, 2019.

The diagnosis of PROM (rupture of membranes) included (1) watery discharge or leakage of amniotic fluid from the cervical os and (2) the pH of the cervicovaginal or vaginal discharge ≥6.5. Gestational age was determined by the last menstruation and ultrasound performed during the first trimester.

### 2.2. Data Collection

The study was approved by the Second Hospital of Shandong University Research Ethics Board (KYLL-2018 (KJ) P-0027). Clinical data were obtained from the electronic medical record of patients with PPROM and their newborns. First, all patients diagnosed with premature rupture of membranes on the first page of medical records from January 1, 2016, to December 31, 2019, were retrieved. Then, patients with rupture of membranes at gestational weeks of 24 to 36^+6^ were retained, and the corresponding neonatal data were retrieved through their mother's name.

### 2.3. Statistical Analysis

The statistical differences of measurement data and enumeration data were tested by sample *t* test and independent chi-square test using SPSS, respectively. A *p* value < 0.05 was considered statistically significant.

### 2.4. Management of PPROM

Patients were counselled by obstetricians about the condition, alternative treatment scheme, and the prognosis of the maternal and newborn at admission. Patients who selected experiment management were given the following treatments. Dexamethasone was given to promote fetal lung maturation (5 mg im bid within a 48 h interval). Antibiotics were applicated prophylactically for seven days at admission. Antibiotics were given again or upgraded when the infection index increased. Magnesium sulfate was applied to protect neonatal nervous system. Ritodrine, nifedipine, or atosiban were used as tocolysis before 35 gestational weeks depending on the patient's status. In addition, the maternal and fetal condition was closely monitored until delivery. Maternal vital signs were monitored every 8 hours. Continuous fetal heart rate monitoring was applicated until delivery. Serum C-reactive protein (CRP), procalcitonin (PCT), and the white blood cell count were checked every other day. Ultrasound was performed once a week to evaluate the status of the fetus. Any abnormal fetal monitoring (fetal movement, amniotic fluid volume, and continuous fetal heart monitoring), maternal complications (clinical chorioamnionitis, continuously rising of infection indicators, and placental abruption), and gestation weeks reached to 35 weeks were indicators for delivery. The mode of delivery depends on the situation of maternal and fetal condition. Pediatricians were informed to participate in the rescue of newborns in advance. Newborns were admitted to neonatal intensive care unit (NICU) according to individual conditions.

## 3. Results

### 3.1. Maternal Characteristics and Maternal and Neonatal Outcomes in Group A

A total of 35 patients were included in this group, including four nulliparous women and six twin-pregnant women. The most common maternal complication was the increased infection index before labour (34.3%), followed by residual fetal membrane (22.9%) and the curettage (17.1%). A total of 41 newborns were born, and more than half of them were abandoned or died (63.41%), nearly a quarter survived (24.39%), and 6 newborns without endotracheal intubation all survived. The most common neonatal complication was neonatal hyperbilirubinemia (27%), followed by neonatal respiratory distress syndrome (24%), neonatal anemia (24%), and neonatal pneumonia (21%) (Table 1).

### 3.2. Maternal Characteristics and Maternal and Neonatal Outcomes in Group B

A total of 88 patients were enrolled in this group, including 12 nulliparous women and 12 twin-pregnant women. Nearly half of the patients delivered by cesarean section (48%), and the highest incidence of maternal complication was increased infection index before labour (36%), followed by pathological placental inflammation (17%), precipitate labor (15%), and fetal distress (15%). There were a total of 94 newborns in this group, of which 82 survived. About four-fifths of the newborns suffered from neonatal pneumonia (81%) and neonatal hyperbilirubinemia (79%), and about half of the newborns were with complicated patent foramen ovale (50%) or electrolyte disorder (48%) (Table 2).

### 3.3. Maternal Characteristics and Maternal and Neonatal Outcomes in Group C

In total, 160 patients were screened for enrollment in group C, including 19 nulliparous women and 17 twin-pregnant women. The most frequent maternal complication was increased infection index before labour (26%), followed by precipitate labor (18%), fever (10%), and fetal distress (10%). Among 177 newborns, only one died. The top three neonatal complications were neonatal pneumonia (77%), neonatal hyperbilirubinemia (82%), and patent foramen ovale (47%) (Table 3).

### 3.4. Maternal Characteristics and Maternal and Neonatal Outcomes in Group D

In group D, 567 patients were reviewed. Among them, 241 were nulliparous, and 33 were twin pregnancy. More than 10% pregnant women were complicated by precipitate labor, and nearly 10% of pregnant women were complicated by fetal distress and increased infection index before labour. The most common complications included neonatal hyperbilirubinemia (44%), neonatal pneumonia (29%), and patent foramen ovale (24%) (Table 4).

### 3.5. Comparison of Maternal and Neonatal Outcomes between B1 Group and B2 Group

According to the median latency period of group B (4 days), the group B was divided into two groups B1 (the latency period ≤4 days, *n* = 48) and B2 (the latency period>4 days, *n* = 46).

In order to compare the maternal outcome, 14 indexes, including cesarean section rate, increased infection index before labour, and fever were observed. It was found that the increased infection index before labour in group B2 was twice as that in group B1 (*p* < 0.05).

To observe neonatal outcomes, we counted all neonatal complications and compared the high incidence rate index between group B1 and group B2. The results showed that the majority of neonatal index in group B2 were better than those in group B1, but only respiratory distress syndrome, electrolyte disturbance, and premature brain were statistically different between two groups. The incidence of respiratory distress syndrome in group B2 was about 1/3 of that in group B1 (B2 VS B1: 13.0% VS 33.3%, *p* = 0.028), and the incidence of electrolyte disorder in group B2 was about half of that in group B1 (B2 VS B1: 34.8% VS 60.4%, *p* = 0.015). The birth weight and Apgar scores (1 min, 5 min) of group B2 (9.09 ± 1.77, 9.80 ± 0.52) were significantly higher than those of group B1 (7.98 ± 2.58, 9.25 ± 1.51), and the difference was statistically significant. The average length of neonatal stay in group B2 (21.70 ± 12.11) was shorter than that in group B1 (25.33 ± 17.18), but the difference was not statistically significant (Table 5).

### 3.6. Comparison of Maternal and Neonatal Outcomes between Group C1 and Group C2

The group C were divided into two groups based on the median latency period (3 days) C1 (the latency period ≤3 days, *n* = 88) and C2 (the latency period >3 days, *n* = 72).

To compare the pregnancy outcome between group C1 and group C2, we reviewed all maternal and neonatal complications and compared indexes with high incidence rate. The maternal results showed the increased infection index before labour in group C2 was more than 4 times as that in group C1 (C2 VS C1: 45.83% VS 10.23%, *p* < 0.05). Neonatal outcome showed that the average birth weight in group C2 was about 200 g higher than that in group C1 (C2 VS C1: 2304.11 ± 369.13 VS 2140.59 ± 355.27, *p* = 0.003), and the average length of neonatal stay in group C2 was about 2 days shorter than that in group C1 (C2 VS C1: 2304.11 ± 369.13 VS 2140.59 ± 355.27, *p* = 0.003). Except that mycotic infection rate of group C2 was 4 times as that of group C1, all the other neonatal complications in group C2 were significantly lower than those in group C1, but there was no statistical difference (Table 6).

## 4. Discussion

PPROM is a serious pregnancy complication responsible for 28% of neonatal morbidities worldwide, which causes one-third of preterm birth [16]. PPROM can be caused by a variety of pathologic mechanisms that act individually or in concert [17, 18]. According to ACOG, antibiotics, single-course of corticosteroids, and vaginal-rectal swab for GBS culture (GBS prophylaxis was administered when necessary) are recommended to patients with PPROM before 34 gestational weeks. In addition, magnesium sulfate was given for neuroprotection before anticipated delivery for pregnancies before 32 gestational weeks [1]. The optimal time for delivery depends on a continuous evaluation of gestational age, maternal and fetal complications, and even the medical service quality level. Previous studies have shown mixed results on the expected treatment results [19, 20]. A meta-analysis of 23 randomized controlled trials (8,615 women) showed that shorter latency period was beneficial to both the mother and newborn [19]. However, short latency period in patients with PPROM between 28 and 34 weeks carries some maternal and neonatal risks with no additional benefits [20].

Current research showed the incidence of all serious neonatal complications was high among patients with gestation age between 28 and 31^+6^ weeks. Prolonged gestational weeks (>4 days) significantly reduced the incidences of neonatal respiratory distress syndrome, premature brain, and electrolyte disorder and meanwhile increased neonatal weight and improved neonatal Apgar score. At the same time, it did not increase the risk of serious maternal complications. These findings were consistent with the previous research results [19, 21]. Reviewing the pregnancy outcomes of patients with gestational weeks at 32–33^+6^ weeks, prolonging gestational weeks not only improved the neonatal birth weight and decreased average length of stay but also significantly increased the risk of maternal infection. This result is inconsistent with previous studies [22]. Accordingly, it is recommended to extend the gestational week for patients with gestational weeks between 28 and 31^+6^ weeks. The analysis of the pregnancy outcome of patients with gestational week between 28 and 31^+6^ weeks showed the incidence rate of all serious neonatal complications was high. Prolonged gestational week of patients with gestation week between 32 and 33^+6^ weeks increased birth weight and shortened neonatal stay, but did not statistically reduce the incidence rate of neonatal complications. The possible reasons are as follows: first, under the current neonatal treatment conditions, while the extension of gestational weeks is of great significance for fetal maturity with gestational week between 28 and 31^+6^, it did not benefit newborns with gestation week greater than 32 weeks. Second is closely monitoring the infection index. Taking persistent increased infection index before labour, rather than chorioamnionitis as the indicator of pregnancy termination, greatly reduces the infection risk of mothers and newborns.

The neonatal mortality rate in 24–27^+6^ weeks was higher than that previously reported [22, 23]. The reason is that more than half of newborns were abandoned before or at birth, as those families gave them up considering the prognosis and treatment cost of newborns. In this group, 10 of the 15 children admitted to NICU (neonatal intensive care unit) finally survived (66.7%), and the six newborns without endotracheal intubation at birth all survived. Perhaps the independence of endotracheal intubation is an indicator of good prognosis of newborns, which requires further studies to confirm. According to the detailed analysis results, obstetricians and pediatrician should give more optimistic suggestion to their parents, especially for newborns who do not need endotracheal intubation at birth.

The contribution of this study lies in patient grouping according to gestational week, which reduced the bias caused by gestational age and the observation of all pregnancy index. The limitation of this study is that the number of patients in some groups is relatively small, and more patients should be recruited for further research.

In conclusion, this study revealed that pregnancy outcome of patients with PPROM were significantly associated with gestational week or the latency period. When the gestational age is 24–27^+6^, the mortality rate of newborns was high because they were abandoned, but the survival rate of newborns who received active treatment reached to 66.7%. The independence of endotracheal intubation was a good indicator of newborn prognosis. Increased infection index before labour was common maternal complication in four groups. Neonatal hyperbilirubinemia and neonatal pneumonia were common neonatal complications in four groups. The prolongation of latency period was beneficial to newborns with gestational week at 28–31^+6^ weeks, while it did not benefit patients with gestation week beyond 32 weeks. These results can guide the clinical treatment to improve the pregnancy outcome of patients with PPROM.

## Figures and Tables

**Table 1:** Clinical outcomes in cases of PPROM (GA 24–27.6).

Characteristics	Result
Number of women with PPROM	35
Maternal age (mean ± S.D.)	32.0 ± 5.1
Weeks of gestation at admission (mean ± S.D.)	26.7 ± 0.78
Maternal age	32.0 ± 5.0
Nulliparous, *n* (%)	4(11.4%)
Pregnancy	
Singleton, *n* (%)	29(82.9%)
Twin, *n* (%)	6(17.1%)

Maternal outcome	
Major maternal complications	
Cesarean delivery, *n* (%)	2(5.7%)
Increased infection index before labour, *n* (%)	12(34.3%)
Fetal membrane residue, *n* (%)	8(22.9%)
Curettage, *n* (%)	6(17.1%)
Pathological placental membrane inflammation, *n* (%)	3(8.6%)

Neonatal outcomes	
Number of theoretical newborns	41
The fetuses were abandoned before birth	4(9.8%)
Number of newborns in the real world	37
Neonatal death/be abandoned at birth, *n* (%)	26(63.4%)
Neonatal survival, *n* (%)	10(24.39%)
Birth weight (mean ± S.D.)	1068 ± 151
NICU admission, *n* (%)	15(40.5%)
Length of hospitalization/d	58.5 ± 15.0

Major neonatal complications	
Neonatal hyperbilirubinemia, *n* (%)	10(27%)
Endotracheal intubation, *n* (%)	9(24%)
Neonatal anemia, *n* (%)	9(24%)
Neonatal respiratory distress syndrome, *n* (%)	9(24%)
Neonatal pneumonia, *n* (%)	8(21%)
Electrolyte disorder, *n* (%)	8(21%)
Bronchopulmonary dysplasia, *n* (%)	7(18%)
Sepsis, *n* (%)	5(13.5%)
Immature retina (double)	5(13.5%)
Neonatal asphyxia, *n* (%)	4(10.8%)
Neonatal hypoglycemia, *n* (%)	3(8.1%)
Neonatal hypoproteinemia, *n* (%)	3(8.1%)
Myocardial damage, *n* (%)	3(8.1%)
Liver damage, *n* (%)	3(8.1%)
Neonatal hypoxic ischemic encephalopathy, *n* (%)	1(2.7%)
Abnormal coagulation function, *n* (%)	1(2.7%)

**Table 2:** Clinical outcomes in cases of PPROM (GA 28–31.6).

Characteristics	Result
Number of women with PPROM	88
Maternal age (mean ± S.D.)	30.4 ± 5.0
Weeks of gestation at admission (mean ± S.D.)	30.2 ± 1.1
Nulliparous, *n* (%)	12,(13.6%)
Pregnancy	
Singleton, *n* (%)	82,(93.18%)
Twin, *n* (%)	6(6.81%)
Latency period (d)	5.9 ± 5.9

Maternal outcome	
Major maternal complications	
Cesarean delivery, *n* (%)	42,(48%)
Increased infection index before labour, *n* (%)	32,(36%)
Pathological placental membrane inflammation, *n* (%)	15,(17%)
Precipitate labor, *n* (%)	13,(15%)
Fetal distress, *n* (%)	13,(15%)
Fever, *n* (%)	8,(9%)
Placental adhesions, *n* (%)	6,(7%)
Prolapse of umbilical cord, *n* (%)	4,(5%)
Uterine atony, *n* (%)	3,(3%)
Fetal membrane residue, *n* (%)	3,(3%)
Placental abruption, *n* (%)	3,(3%)
Postpartum hemorrhage, *n* (%)	2,(2%)
Chorioamnionitis, *n* (%)	2,(2%)
Curettage, *n* (%)	2,(2%)

Neonatal outcomes	
Neonatal number	94
Neonatal death/be abandoned, *n* (%)	12,(13%)
Neonatal survival, *n* (%)	82,(87%)
Birth weight/g (mean ± S.D.)	1687.2 ± 373.5
Apgar score at 1 minute	8.5 ± 2.3
Apgar score at 5 minutes	9.6 ± 1.2
Hospitalization length (d)	23.1 ± 15.1
Hospitalization length of survival (d)	26.0 ± 14.0
Endotracheal intubation, *n* (%)	16,(17%)
NICU admission, *n* (%)	89,(95%)

Major neonatal condition	
Neonatal pneumonia, *n* (%)	76,(81%)
Neonatal hyperbilirubinemia, *n* (%)	74,(79%)
Patent foramen ovale, *n* (%)	47,(50%)
Electrolyte disorder, *n* (%)	45,(48%)
Neonatal anemia, *n* (%)	32,(34%)
Premature brain, *n* (%)	26,(28%)
Neonatal asphyxia, *n* (%)	24,(26%)
Myocardial damage, *n* (%)	23,(24%)
Neonatal respiratory distress syndrome, *n* (%)	22,(23%)
Neonatal hypoglycemia, *n* (%)	20,(21%)
Patent ductus arteriosus, *n* (%)	19,(20%)
Sepsis, *n* (%)	28,(30%)
Neonatal hypoproteinemia, *n* (%)	16,(17%)
ABO hemolytic disease of newborn, *n* (%)	11,(12%)
Abnormal coagulation function, *n* (%)	11,(12%)
Immature retina (double), *n* (%)	11,(12%)
High TSH/hypothyroidism, *n* (%)	11,(12%)
Mycotic infection, *n* (%)	9,(10%)
Neonatal intracranial hemorrhage, *n* (%)	9,(10%)
Neonatal hypoxic ischemic encephalopathy, *n* (%)	6,(6%)
Neonatal respiratory failure, *n* (%)	5,(5%)
Pulmonary hypertension, *n* (%)	5,(5%)
Bronchopulmonary dysplasia, *n* (%)	4,(4%)
Ureaplasma urealyticum infection, *n* (%)	4,(4%)
Neonatal conjunctivitis, *n* (%)	4,(4%)
Neonatal meningitis, *n* (%)	3,(3%)
Neonatal thrombocytopenia, *n* (%)	3,(3%)
Neonatal necrotizing colitis, *n* (%)	3,(3%)
Cholestasis, *n* (%)	3,(3%)

**Table 3:** Clinical outcomes in cases of PPROM (GA 32–33.6).

Characteristics	Result
Number of women with PPROM	160
Maternal age (mean ± S.D.)	30.5 ± 5.3
Weeks of gestation at admission (mean ± S.D.)	32.9 ± 0.51
Nulliparous, *n* (%)	19 (11.87%)
Pregnancy	
Singleton, *n* (%)	142 (88.8%)
Twin, *n* (%)	17 (10.63%)
Latency period (d)	4.0 ± 3.9

Maternal outcome	
Major maternal complications	
Cesarean delivery, *n* (%)	74,(46%)
Increased infection index before labour, *n* (%)	42,(26%)
Precipitate labor, *n* (%)	29,(18%)
Fever, *n* (%)	16,(10%)
Fetal distress, *n* (%)	12,(8%)
Pathological placental membrane inflammation, *n* (%)	11,(7%)
Placental adhesions, *n* (%)	7,(4%)
Uterine atony, *n* (%)	6,(4%)
Postpartum hemorrhage, *n* (%)	6,(4%)
Fetal membrane residue, *n* (%)	6,(4%)
Curettage, *n* (%)	4,(3%)
Placental abruption, *n* (%)	4,(3%)
Chorioamnionitis, *n* (%)	2,(1%)
Prolapse of umbilical cord, *n* (%)	1,(1%)

Neonatal outcomes	
Neonatal number	177
Neonatal death/be abandoned, *n* (%)	1,(1%)
Neonatal survival, *n* (%)	176,(99%)
Birth weight/g (mean ± S.D.)	2210.3 ± 367.6
Apgar score at 1 minute	9.5 ± 1.1
Apgar score at 5 minute	9.8 ± 0.6
Hospitalization length (d)	11.4 ± 7.1
Hospitalization length of survival (d)	11.4 ± 7.1
Endotracheal intubation, *n* (%)	7,(4%)
NICU admission, *n* (%)	165,(93%)

Major neonatal condition	
Neonatal hyperbilirubinemia, *n* (%)	145,(82%)
Neonatal pneumonia, *n* (%)	136,(77%)
Patent foramen ovale, *n* (%)	83,(47%)
Neonatal hypoglycemia, *n* (%)	49,(28%)
Myocardial damage, *n* (%)	42,(24%)
Patent ductus arteriosus, *n* (%)	32,(18%)
Electrolyte disorder, *n* (%)	31,(18%)
Premature brain, *n* (%)	24,(14%)
Neonatal anemia, *n* (%)	22,(12%)
Pulmonary hypertension, *n* (%)	19,(11%)
Sepsis, *n* (%)	25,(14%)
Neonatal asphyxia, *n* (%)	13,(7%)
Neonatal intracranial hemorrhage, *n* (%)	13,(7%)
Neonatal hypoproteinemia, *n* (%)	11,(6%)
Atrial septal defect, *n* (%)	11,(6%)
ABO hemolytic disease of newborn, *n* (%)	10,(6%)
Neonatal respiratory distress syndrome, *n* (%)	10,(6%)
Neonatal hypoxic ischemic encephalopathy, *n* (%)	7,(4%)
Abnormal coagulation function, *n* (%)	7,(4%)
Ventricular septal defect, *n* (%)	6,(3%)
Mycotic infection, *n* (%)	5,(3%)
Immature retina (double), *n* (%)	5,(3%)
Neonatal thrombocytopenia, *n* (%)	4,(2%)
Neonatal gastrointestinal bleeding, *n* (%)	4,(2%)
Neonatal respiratory failure, *n* (%)	4,(2%)
Neonatal meningitis, *n* (%)	3,(2%)
Septic shock, *n* (%)	1,(1%)

**Table 4:** Clinical outcomes in cases of PPROM (GA 34–36.6).

Characteristics	Result
Number of women with PPROM	567
Maternal age (mean ± S.D.)	30.66 ± 4.98
Weeks of gestation at admission (mean ± S.D.)	35.64 ± 0.83
Nulliparous, *n* (%)	241,(42.5%)
Pregnancy	
Singleton, *n* (%)	530,(93.4%)
Twin, *n* (%)	33(5.82%)
Latency period (d)	0.88 ± 1.68

Maternal outcome	
Major maternal complications	
Cesarean delivery, *n* (%)	284,(50%)
Precipitate labor, *n* (%)	78,(14%)
Fetal distress, *n* (%)	48,(8%)
Increased infection index before labour, *n* (%)	37,(7%)
Fever, *n* (%)	29,(5%)
Uterine atony, *n* (%)	25,(4%)
Postpartum hemorrhage, *n* (%)	15,(3%)
Placental abruption, *n* (%)	12,(2%)
Pathological placental membrane inflammation, *n* (%)	10,(2%)
Placental adhesions, *n* (%)	7,(1%)
Curettage, *n* (%)	6,(1%)
Fetal membrane residue, *n* (%)	3,(1%)
Prolapse of umbilical cord, *n* (%)	2,(0%)
Chorioamnionitis, *n* (%)	1,(0%)

Neonatal outcomes	
Neonatal number	600
Neonatal death/be abandoned, *n* (%)	2,(0%)
Neonatal survival, *n* (%)	598,(100%)
Birth weight/g(mean ± S.D.)	2706.89 ± 414.28
Apgar score at 1 minute	9.88 ± 0.64
Apgar score at 5 minute	9.96 ± 0.36
Hospitalization length (d)	4.52 ± 5.66
Endotracheal intubation, *n* (%)	3,(1%)
NICU admission, *n* (%)	327,(55%)
Major neonatal condition	
Neonatal hyperbilirubinemia, *n* (%)	264,(44%)
Neonatal pneumonia, *n* (%)	176,(29%)
Patent foramen ovale, *n* (%)	144,(24%)
Neonatal hypoglycemia, *n* (%)	80,(13%)
Myocardial damage, *n* (%)	69,(12%)
Neonatal infection	55,(9%)
Patent ductus arteriosus, *n* (%)	45,(8%)
Electrolyte disorder, *n* (%)	41,(7%)
ABO hemolytic disease of newborn, *n* (%)	35,(6%)
Pulmonary hypertension, *n* (%)	27,(5%)
Atrial septal defect, *n* (%)	20,(3%)
Premature brain, *n* (%)	19,(3%)
Neonatal anemia, *n* (%)	16,(3%)
Septicemia, *n* (%)	24,(4%)
Neonatal intracranial hemorrhage, *n* (%)	11,(2%)
Ventricular septal defect, *n* (%)	10,(2%)
Neonatal asphyxia, *n* (%)	8,(1%)
Neonatal respiratory distress syndrome, *n* (%)	8,(1%)
Abnormal coagulation function, *n* (%)	6,(1%)
Neonatal respiratory failure, *n* (%)	7,(1%)

**Table 5:** Comparison of maternal and neonatal outcomes between B1 group and B2 group.

Comparison of maternal outcomes	Latency period ≤4 (*n* = 45)	Latency period ＞4 (*n* = 43)	*p* value (chi- square test/*t*-test)

Cesarean delivery, *n* (%)	17,(37.8%)	21,(48.8%)	0.39
Precipitate labor	7,(15.6%)	8,(18.6%)	1
Increased infection index before labour (%)	11,(24.44%)	21,(48.84%)	0.026
Pathological placental membrane inflammation (%)	5,(11.1%)	8,(19%)	0.158
Fetal distress, *n* (%)	4,(8.9%)	8,(19%)	0.14
Fever, *n* (%)	3,(6.7%)	10,(23%)	0.429
Placental adhesions, *n* (%)	2,(4.4%)	3,(7%)	0.479
Prolapse of umbilical cord, *n* (%)	2,(4.4%)	2,(5%)	1
Uterine atony, *n* (%)	2,(4.4%)	1,(2%)	1
Fetal membrane residue, *n* (%)	2,(4.4%)	2,(5%)	1
Placental abruption, *n* (%)	3,(6.7%)	0,(0%)	0.242
Postpartum hemorrhage, *n* (%)	1,(2.2%)	1,(2%)	1
Chorioamnionitis, *n* (%)	1,(2.2%)	0,(0%)	1
Curettage, *n* (%)	1,(2.2%)	1,(2%)	1

Comparison of neonatal outcomes	Latency period ≤4(*n* = 48)	Latency period ＞4(*n* = 46)	*p* value (chi-square test/*t*-test)

Birth weight/g (mean ± S.D.)	1548.96 ± 344.51	1830.65 ± 347.16	<0.01
Apgar score at 1 minute	7.98 ± 2.58	9.09 ± 1.77	0.018
Apgar score at 5 minutes	9.25 ± 1.51	9.80 ± 0.52	0.027
Hospitalization length (d)	25.33 ± 17.18	21.70 ± 12.11	0.249
Neonatal death/be abandoned, *n* (%)	9,(18.8%)	3,(6.5%)	0.121
Neonatal survival, *n* (%)	39,(81.3%)	43,(93.5%)	0.121
Endotracheal intubation, *n* (%)	11,(22.9%)	5,(10.9%)	0.173
NICU admission, *n* (%)	45,(93.8%)	44,(95.7%)	1
Neonatal pneumonia, *n* (%)	40,(83.3%)	36,(78.3%)	0.605
Neonatal hyperbilirubinemia, *n* (%)	36,(75.0%)	38,(82.6%)	0.453
Patent foramen ovale, *n* (%)	23,(47.9%)	20,(43.5%)	0.837
Electrolyte disorder, *n* (%)	29,(60.4%)	16,(34.8%)	0.015
Neonatal anemia, *n* (%)	20,(41.7%)	12,(26.1%)	0.131
Premature brain, *n* (%)	14,(29.2%)	12,(26.1%)	0.002
Neonatal asphyxia, *n* (%)	15,(31.3%)	9,(19.6%)	0.24
Myocardial damage, *n* (%)	11,(22.9%)	12,(26.1%)	0.812
Neonatal respiratory distress syndrome, *n* (%)	16,(33.3%)	6,(13.0%)	0.028
Neonatal hypoglycemia, *n* (%)	8,(16.7%)	10,(21.7%)	0.318
Patent ductus arteriosus, *n* (%)	9,(18.8%)	14,(30.4%)	0.8
Sepsis, *n* (%)	9,(18.8%)	7,(15.2%)	0.264
Neonatal hypoproteinemia, *n* (%)	10,(20.8%)	6,(13.0%)	0.413
ABO hemolytic disease of newborn, *n* (%)	6,(12.5%)	5,(10.9%)	1
Abnormal coagulation function, *n* (%)	5,(10.4%)	6,(13.0%)	0.756
Immature retina (double), *n* (%)	7,(14.6%)	4,(8.7%)	0.524
Mycotic infection, *n* (%)	5,(10.4%)	4,(8.7%)	1
Neonatal intracranial hemorrhage, *n* (%)	7,(14.6%)	2,(4.3%)	0.159
Neonatal hypoxic ischemic encephalopathy, *n* (%)	4,(8.3%)	2,(4.3%)	0.678
Neonatal respiratory failure, *n* (%)	2,(4.2%)	3,(6.5%)	0.674
Pulmonary hypertension, *n* (%)	4,(8.3%)	1,(2.2%)	0.362
Bronchopulmonary dysplasia, *n* (%)	4,(8.3%)	0,(0.0%)	0.117
Ureaplasma urealyticum infection, *n* (%)	3,(6.3%)	1,(2.2%)	0.617
Neonatal conjunctivitis, *n* (%)	3,(6.3%)	1,(2.2%)	0.617
Neonatal meningitis, *n* (%)	3,(6.3%)	0,(0.0%)	0.242
Neonatal thrombocytopenia, *n* (%)	3,(6.3%)	0,(0.0%)	0.242
Neonatal necrotizing colitis, *n* (%)	2,(4.2%)	0,(0.0%)	1

**Table 6:** Comparison of maternal and neonatal outcomes between C1 group and C2 group.

Comparison of maternal outcomes	Latency period ≤3 (*n* = 88)	Latency period ＞3 (*n* = 72)	*p* value (chi-square test/*t*-test)
Cesarean delivery, *n* (%)	38,(43.2%)	36,(50.0%)	0.428
Precipitate labor	21,(23.9%)	8,(11.1%)	0.041
Increased infection index before labour(%)	9,(10.23%)	33,(45.83%)	<0.01
Fever, *n* (%)	7,(8.0%)	7,(10%)	0.201
Pathological placental membrane inflammation (%)	6,(6.8%)	5,(7%)	1
Fetal distress, *n* (%)	5,(5.7%)	7,(10%)	0.378
Uterine atony, *n* (%)	5,(5.7%)	1,(1%)	0.224
Postpartum hemorrhage, *n* (%)	4,(4.5%)	2,(3%)	0.691
Placental adhesions, *n* (%)	3,(3.4%)	4,(6%)	0.702
Placental abruption, *n* (%)	3,(3.4%)	1,(1%)	0.628
Fetal membrane residue, *n* (%)	2,(2.3%)	4,(6%)	0.41
Curettage, *n* (%)	2,(2.3%)	2,(3%)	1
Prolapse of umbilical cord, *n* (%)	1,(1.1%)	0,(0%)	1
Chorioamnionitis, *n* (%)			0.201

Comparison of neonatal outcomes	Latency period≤3(*n* = 104)	Latency period＞3(*n* = 73)	*p* value (chi-square test/*t*-test)

Birth weight/g(mean ± S.D.)	2140.59 ± 355.27	2304.11 ± 369.13	0.003
Apgar score at 1 minute	9.47 ± 1.39	9.60 ± 0.83	0.47
Apgar score at 5 minute	9.85 ± 0.62	9.82 ± 0.59	0.77
Hospitalization length/d	12.37 ± 7.67	10.11 ± 5.99	0.037
Neonatal death/be abandoned, *n* (%)	1,(0.96%)	0,(0.00%)	1
Neonatal survival, *n* (%)	103,(99.04%)	73,(100.00%)	1
NICU admission, *n* (%)	97,(93.27%)	49,(67.12%)	1
Neonatal hyperbilirubinemia, *n* (%)	85,(81.73%)	44,(60.27%)	1
Neonatal pneumonia, *n* (%)	77,(74.04%)	44,(60.27%)	0.366
Patent foramen ovale, *n* (%)	48,(46.15%)	30,(41.10%)	0.879
Neonatal hypoglycemia, *n* (%)	31,(29.81%)	13,(17.81%)	0.498
Patent ductus arteriosus, *n* (%)	23,(22.12%)	9,(12.33%)	0.114
Electrolyte disorder, *n* (%)	21,(20.19%)	7,(9.59%)	0.318
Premature brain, *n* (%)	17,(16.35%)	4,(5.48%)	0.265
Neonatal anemia, *n* (%)	16,(15.38%)	4,(5.48%)	0.173
Pulmonary hypertension, *n* (%)	13,(12.50%)	5,(6.85%)	0.463
Sepsis, *n* (%)	18,(17.31%)	5,(6.85%)	0.19
Neonatal asphyxia, *n* (%)	8,(7.69%)	4,(5.48%)	1
Neonatal intracranial hemorrhage, *n* (%)	8,(7.69%)	4,(5.48%)	1
Neonatal hypoproteinemia, *n* (%)	7,(6.73%)	3,(4.11%)	0.766
Atrial septal defect, *n* (%)	9,(8.65%)	2,(2.74%)	1
ABO hemolytic disease of newborn, *n* (%)	6,(5.77%)	2,(2.74%)	1
Neonatal respiratory distress syndrome, *n* (%)	8,(7.69%)	1,(1.37%)	0.2
Neonatal hypoxic ischemic encephalopathy, *n* (%)	5,(4.81%)	2,(2.74%)	0.701
Abnormal coagulation function, *n* (%)	4,(3.85%)	2,(2.74%)	1
Ventricular septal defect, *n* (%)	4,(3.85%)	2,(2.74%)	1
Myocardial damage, *n* (%)	26,(25.00%)	12,(16.44%)	0.721
Immature retina (double), *n* (%)	4,(3.85%)	0,(0.00%)	0.406
Neonatal thrombocytopenia, *n* (%)	2,(1.92%)	1,(1.37%)	1
Neonatal respiratory failure, *n* (%)	3,(2.88%)	1,(1.37%)	0.644
Neonatal meningitis, *n* (%)	2,(1.92%)	0,(0.00%)	1
Septic shock, *n* (%)	1,(0.96%)	0,(0.00%)	1
Endotracheal intubation, *n* (%)	6,(5.77%)	1,(1.37%)	0.242
Mycotic infection	4,(3.85%)	12,(16.44%)	0.406
Bronchopulmonary dysplasia	1,(0.96%)	0,(0.00%)	1
Ureaplasma urealyticum infection	1,(0.96%)	0,(0.00%)	1

## Data Availability

No datasets were generated or analysed during the current study.

## References

[1] Siegler Y., Weiner Z., Solt I. (2020). Prelabor rupture of membranes: ACOG practice bulletin, number 217. *Obstetrics & Gynecology*.

[2] Thomson A. J. (2019). Care of women presenting with suspected preterm prelabour rupture of membranes from 24(+0) weeks of gestation: green-top guideline No. 73. *Bjog*.

[3] Ananth C. V., Oyelese Y., Srinivas N., Yeo L., Vintzileos A. M. (2004). Preterm premature rupture of membranes, intrauterine infection, and oligohydramnios. *Obstetrics & Gynecology*.

[4] Stoll B. J., Hansen N. I., Bell E. F. (2010). Neonatal outcomes of extremely preterm infants from the NICHD Neonatal Research Network. *Pediatrics*.

[5] Hackney D. N., Kuo K., Petersen R. J., Lappen J. R. (2016). Determinants of the competing outcomes of intrauterine infection, abruption, or spontaneous preterm birth after preterm premature rupture of membranes. *Journal of Maternal-Fetal and Neonatal Medicine*.

[6] Menon R., Fortunato S. J. (2007). Infection and the role of inflammation in preterm premature rupture of the membranes. *Best Practice & Research Clinical Obstetrics & Gynaecology*.

[7] Fortunato S. J., Menon R., Bryant C., Lombardi S. J. (2000). Programmed cell death (apoptosis) as a possible pathway to metalloproteinase activation and fetal membrane degradation in premature rupture of membranes. *American Journal of Obstetrics and Gynecology*.

[8] Menon R., Richardson L. S. (2017). Preterm prelabor rupture of the membranes: A disease of the fetal membranes. *Seminars in Perinatology*.

[9] Weisz B., David A. L., Chitty L. (2008). Association of isolated short femur in the mid-trimester fetus with perinatal outcome. *Ultrasound in Obstetrics and Gynecology*.

[10] Gejo N. G., W/mariam M. T., Kebede B. A. (2021). Factors associated with preterm birth at Wachemo University Nigist Eleni Mohammed memorial hospital, southern Ethiopia: Case-control study. *BMC Pregnancy and Childbirth*.

[11] Waters T. P., Mercer B. (2011). Preterm PROM. *Clinical Obstetrics and Gynecology*.

[12] González-Mesa E., Blasco-Alonso M. (2021). Obstetric and perinatal outcomes after very early preterm premature rupture of membranes (PPROM)-A retrospective analysis over the period 2000-2020. *Medicina*.

[13] Roberts C. L., Wagland P., Torvaldsen S., Bowen J. R., Bentley J. P., Morris J. M. (2017). Childhood outcomes following preterm prelabor rupture of the membranes (PPROM): A population-based record linkage cohort study. *Journal of Perinatology*.

[14] Sheibani L., Fong A., Henry D. E. (2017). Maternal and neonatal outcomes after antenatal corticosteroid administration for PPROM at 32 to 33 6/7 weeks gestational age(). *Journal of Maternal-Fetal and Neonatal Medicine*.

[15] Subramaniam A., Cliver S. S., Smeltzer S., Tita A. T., Wetta L. L. (2016). Preterm premature rupture of membranes (PPROM): Outcomes of delivery at 32°/7-336/7weeks after confirmed fetal lung maturity (FLM) versus expectant management until 34°/7weeks. *Journal of Maternal-Fetal and Neonatal Medicine*.

[16] Menon R. (2008). Spontaneous preterm birth, a clinical dilemma: etiologic, pathophysiologic and genetic heterogeneities and racial disparity. *Acta Obstetricia et Gynecologica Scandinavica*.

[17] Moore R. M., Mansour J. M, Redline R. W, Mercer B. M, Moore J. J (2006). The physiology of fetal membrane rupture: insight gained from the determination of physical properties. *Placenta*.

[18] Mercer B. (2003). Preterm premature rupture of the membranes. *Obstetrics & Gynecology*.

[19] Middleton P., Shepherd E, Flenady V, McBain R. D, Crowther C. A (2017). Planned early birth versus expectant management (waiting) for prelabour rupture of membranes at term (37 weeks or more). *Cochrane Database of Systematic Reviews*.

[20] Al-Mandeel H., Alhindi M. Y., Sauve R. (2013). Effects of intentional delivery on maternal and neonatal outcomes in pregnancies with preterm prelabour rupture of membranes between 28 and 34 weeks of gestation: A systematic review and meta-analysis. *Journal of Maternal-Fetal and Neonatal Medicine*.

[21] Bond D. M., Middleton P, Levett K. M (2017). Planned early birth versus expectant management for women with preterm prelabour rupture of membranes prior to 37 weeks’ gestation for improving pregnancy outcome. *Cochrane Database of Systematic Reviews*.

[22] Yu H., Wang X., Gao H., You Y., Xing A. (2015). Perinatal outcomes of pregnancies complicated by preterm premature rupture of the membranes before 34 weeks of gestation in a tertiary center in China: A retrospective review. *BioScience Trends*.

[23] Gezer A., Parafit-Yalciner E., Guralp O., Yedigoz V., Altinok T., Madazli R. (2013). Neonatal morbidity mortality outcomes in pre-term premature rupture of membranes. *Journal of Obstetrics and Gynaecology*.

